# Rbm46 regulates mouse embryonic stem cell differentiation by targeting *β-Catenin* mRNA for degradation

**DOI:** 10.1371/journal.pone.0172420

**Published:** 2017-02-17

**Authors:** Lei Zhai, Chenchen Wang, Yuanfan Chen, Shixin Zhou, Lingsong Li

**Affiliations:** 1 Department of Cell Biology, School of Basic Medical Sciences, Peking University Health Science Center, Beijing, China; 2 Peking University Stem Cell Research Center, China National Center for International Research, Peking University Health Science Center, Beijing, China; 3 SARI Center for Stem Cell and Nanomedicine, Shanghai Advanced Research Institute, University of Chinese Academy of Sciences, Shanghai, China; University of Texas at Austin Dell Medical School, UNITED STATES

## Abstract

Embryonic stem cells (ESCs) are pluripotent cells and have the capability for differentiation into any of the three embryonic germ layers. The Wnt/*β-Catenin* pathway has been shown to play an essential role in ESC differentiation regulation. Activation of *β-Catenin* by post-translational modification has been extensively studied. However, mechanism(s) of post-transcriptional regulation of *β-Catenin* are not well defined. In this study, we report an RNA recognition motif-containing protein (RNA binding motif protein 46, RBM46) which regulates the degradation of *β-Catenin* mRNA. Our results show that Rbm46 is distributed primarily in the cytoplasm of mouse ESCs (mESCs) and is elevated during the process of ESC differentiation. In addition, overexpression of Rbm46 results in differentiation of mESCs into trophectoderm, while knock-down of *Rbm46* leads to mESC differentiation into endoderm. β-Catenin, a key effector in the Wnt pathway which has been reported to play a significant role in the regulation of ESC differentiation, is post-transcriptionally regulated by Rbm46. Our study reveals Rbm46 plays a novel role in the regulation of ESC differentiation.

## Introduction

Mouse ESCs (mESCs) were first isolated from the inner cell masses of late blastocysts [1]. These pluripotent cells were found to have potential for differentiation into a wide variety of cell types, and further study showed that mESCs have the capability to differentiate into any of the three embryonic germ layers [2]. Stem cell differentiation is regulated by a complex network which includes certain critical transcription factors such as Nanog, SOX2, and OCT4 [3]. These proteins form a mutual regulatory circuit, and coordinate their activity with other differentiation related transcription factors such as REST, SKIL and HESX1, and with some histone modifying complexes (for example SMARCAD1, MYST3 and SET) [4, 5] to regulate stem cell Differentiation. In addition to this primary regulatory circuit, some signaling pathways are also involved in stem cell regulation [6, 7]. The Wnt signaling pathway has emerged as an essential regulator of stem cells, and over-activation of Wnt signaling is involved in tumorigenesis associated with dysregulation of stem cell self-renewal [8, 9].

Aberration of this transcriptional regulatory circuity, especially the aberration of the Wnt/ β-Catenin/Oct4 pathway may lead to changes in the state of ESC pluripotency which results in an increased tendency for differentiation. Oct4 is involved in the regulation of cell growth and differentiation in a wide variety of tissues and is typically expressed in pluripotent cells of developing embryos [10]. Genome-wide chromatin immunoprecipitation (ChIP) experiments showed that Oct4 binds to a wide variety of downstream target genes essential for self-renewal in each mESC and hESC [11]. The OCT4 protein level determines the differentiation direction of ESC. The critical amount of Oct4 is essential for sustaining ES cell pluripotency, and up or downregulation of Oct4 induces divergent differentiation direction. When the OCT4 protein level reaches a level 2 fold of normal, stem cells are more likely to differentiate into endoderm. However, if the OCT4 level drops to half of its normal value, stem cells differentiate into trophectoderm [12]. In addition, inhibition of the LIF/STAT3 pathway results in differentiation of stem cells into trophectoderm, and low concentrations of LIF and Wnt proteins block ESC differentiation [13]. Inhibition of GSK-3β activity leads to activation of the Wnt pathway and subsequent increase in *β-Catenin* mRNA, thereby promoting the transcription of *Oct4*, *Rex1* and *Nanog* and ultimate change in ESC pluripotency [14–16]. These findings suggest that regulation of β-Catenin by the Wnt pathway is essential for ESC differentiation regulation. It is not known whether *β-Catenin* is also regulated by mechanisms independent of the Wnt pathway in the course of ESC development such as post-transcriptional regulation.

In this study, we report a RNA recognition motif (RRM) containing protein (or RNA binding protein, RBP) referred to as RBM46 which is highly expressed in hESCs. RRM is one of the most abundant protein domains in eukaryotes and is involved in all post-transcriptional events including pre-mRNA processing, splicing, and mRNA editing [17]. Some of the RRM family proteins function in regulation of differentiation in ESCs, central nervous system (CNS) stem cells and progenitor germ cells (PGCs) [18–20]. However, the precise mechanism by which ESC differentiation is regulated is poorly understood. In this study, we reveal a novel Rbm46 function and uncovers a previously undescribed mechanism through which ESC differentiation is regulated by RRM protein.

## Materials and methods

### Cell culture

E14Tg2a mouse ESCs were cultured in the DMEM supplemented with 15% (v/v) fetal calf serum (FCS; Hyclone, Logan, UT, www.hyclone.com), 100 mM 2- mercaptoethanol (Sigma; Cat. No. M7522), nonessential amino acids (Gibco), 2 mM l-glutamine (Chemicon), 1 mM sodium pyruvate (Sigma), and 100 U/mL leukemia inhibitory factor (LIF). Plates were fixed and stained for alkaline phosphatase (Sigma; Cat. No. 86R-1KT) according to the manufacturer’s protocol.

### Western blot analysis and Flag immunoprecipitation

Cells were lysed with lysis buffer (20 mM Tris–HCl, pH 7.5, 150 mM NaCl, 0.5% Triton X-100, 12.5 mM b-glycerophosphate, 1.5 mM MgCl2, 2 mM ethylene glycol tetraacetic acid, 10 mM NaF, and 1 mM Na3VO4) containing protease inhibitors (Roche). Western blot was performed by standard procedures; primary antibodies used in this study: anti-Oct4 (Santa Cruz, sc-365509), anti-Rbm46 (sigma, HPA050601), beta-Actin (santa cruz, sc-47778), Pabpc1 (AVIVA, OAAB01699), GSK-3 (Millipore, 05–412), SSEA-1(Millipore, FCMAB117P). Proteins were visualized with an Odyssey Two-Color Infrared Imaging System (LI-COR Biosciences) according to the manufacturer’s instructions. For Flag immunoprecipitaion, Flag M2 beads (Sigma, F1804) were utilized according to the manufacturer’s protocal.

### Plasmids

Full-length Mouse Rbm46 coding sequence was amplified from mouse testis mRNA and cloned into the pPyCAGIP vector with the following primers: 5’-ATCGCG CTCGAGATGGACTACAAGGACGACGATGACAAGATGAATGAAGAAAACACTGATGGTAC-3’ and 5’-ATATG CGGCCGCTCAGAAGAATGAGGCCTGATTG-3’. Nucleotides targeting the firefly luciferase gene, which has no homology with mouse transcriptome, served as control short hairpin RNA (shRNA). The RNAi oligonucle- otides sequences used are as follows: Rbm46 (siRbm46): 5’- TCCAACAATATCACTTGCTATTCATAGAGATAGCAAGTGATATTGTTGGTTTTTTC-3’. All constructs were verified by sequencing. To generate overexpression or knock- down cells, E14Tg2a ESCs were transfected separately with pPyCAGIP or shRNA constructs using Lipofectamine 2000 and 1 mg/mL of puromycin was added at 48 h post- transfection. About 10 days later, stably transfected cells were expanded and then stored for further analysis.

### Teratocarcinoma formation assay

For teratocarcinoma formation assay, pPE-E14, pPy-RBM46-E14, Non silence-pPE-E14, Rbm46 shRNA-pPE-E14 cells were cultured and suspended at 1 x 10^6^ cells/ml in phosphate-buffered saline (PBS). A total of 100μl of the cell suspension (1 × 10^6^ cells) was subcutaneously injected into the inside of the lower limbs of nude mice purchased from Beijing Vital River Laboratory Animal Technology Co., Ltd. For pPE-E14 and pPy-RBM46-E14 cell lines, seven mice were injected per cell line. For *Non silence*-pPE-E14 and *Rbm46 shRNA*-pPE-E14 cell lines, nine mice were injected per cell line. The transplanted animals were observed routinely every 3–5 days, and tumour growth was measured with a calliper every 3–5 days. The health condition of the mice were monitored and abnormal change in temperature, respiration, feeding behaviour and weight loss was considered as unhealthy signs and the mice would be euthanized. Carbon dioxide was utilized for euthanasia for all the animals. In this study, no mice became ill or died before the experimental endpoint. After 6 weeks post the transplantation, tumours were isolated from the mice. Animals were humanely sacrificed prior to teratocarcinoma isolation. The sacrificed animals were subjected to general inspection. The teratocarcinoma samples were then weighed and subjected to RT-PCR analysis. All mice used in the study were bred and maintained at the Experimental Animal Center, Peking University Health Sciences Center (Beijing, China). The animal experiment protocol was approved by the Biomedical Research Ethics Committee of Peking University and strictly adhered to the American Physiological Society’s “Guiding Principles in the Care and Use of Vertebrate Animals in Research and Training”.

### RNA immunoprecipitation

For the RNA-IP assay, empty vector of FLAG-Rbm46 was transfected into E14 cells for 48 hours. The cells were collected and subsequently lysed with lysis buffer (20 mM Tris–HCl, pH 7.5, 150 mM NaCl, 0.5% Triton X-100, 12.5 mM b-glycerophosphate, 1.5 mM MgCl_2_, 2 mM ethylene glycol tetraacetic acid, 10 mM NaF, and 1 mM Na_3_VO_4_) containing protease inhibitors (Roche). Followed by a FLAG immunoprecipitation using FLAG M2 beads (Sigma, F1804). The beads were washed and eluted with 0.1M Glycine, pH 3.0 and neutralized with 1M Tris-HCl, pH 8.0. The eluate was used for RNA extraction using Trizole reagent (Invitrogen), followed by RT-PCR to detect *beta-catenin* and *gapdh*. Primers are listed in S1 Table.

### RT-PCR analysis

RNA was isolated using Trizol (Invitrogen). Reverse transcriptase (Promega) was utilized for cDNA synthesis. Real-time polymerase chain reaction (PCR) was carried out on the SYBR Premix Ex Taq II detection system (Takara) using SYBR dye. The amount of mRNA level was determined by the ΔΔCt method. Primers are listed in S1 Table.

### Immunofluorescence microscopy

Cells on coverslips were fixed in cold methanol for 15min. And were then washed in phosphate-buffered saline (PBS) for three times, cells were subsequently blocked in PBS containing 5% BSA for 30min and then incubated with mouse or rabbit primary antibodies in PBS containing 2.5% BSA for 2–12 h at 37°C. After three washes, cells were incubated with fluorescein isothiocyanate-conjugated a-mouse and PE- conjugated a-rabbit secondary antibodies for 1 h at 37°C and then with 4, 6-diamidino-2-phenylindole (Roche) for 15 min. The coverslips were washed extensively and mounted onto slides. Imaging of the cells was carried out using the Zeiss LSM 510 Meta Confocal Microscope.

### Flow cytometry

One million cultured cells per sample were dissociated with 0.25% trypsin (Gibco; Cat. No. 25200–056). Cells were then resuspended in 1:3 volumes of ice-cold PBS and 100% ethanol and then incubated on ice for 30 min. After centrifugation, the cell pellet was washed 3 times with PBS and centrifuged for 5 min. Cells were then incubated in the dark in 1 mL PBS containing RNase (12.5 g/mL; Tiangen) for 30 min and propidium iodide (3 g/mL; Sigma) and analyzed by flow cytometry. Analyses were performed by flow cytometry (FACS Calibur; BD Biosciences) using CellQuest software (BD Biosciences) and the ModFit software (Verity Software House).

### Statistical analysis

The statistical significance of the mean differences between two samples was analysed by the Student two-tailed t test. To compare means of more than three samples, One-way ANOVA with Tukey’s post hoc test was used for analysis. Data are shown as means ± SD of the results of at least three independent experiments. Values of p < 0.05 were considered significant.

## Results

### Rbm46 is elevated during mESC differentiation

In our preliminary study, we found that RBM46 is highly expressed in hESC (data not shown). Given that RRM proteins are essential for early embryo development [17], we hypothesized RBM46 may regulate certain genes critical for ESC differentiation. RBM46 is highly conserved in various species, suggesting it has significant biological function (S1A Fig). Bioinformatics indicate RBM46 contains three RRM domains which are located at aa 62–135, aa 142–219 and aa 237–304 (S1B Fig). We first evaluated the influence of RBM46 on ESC proliferation. To this end, FLAG-Rbm46 plasmid was transfected into E14/T mESCs to establish cell lines able to stably express FLAG-Rbm46 (pPy-Rbm46-E14) or empty vector (pPE-E14 (Fig 1A). A colony formation assay showed that pPy-Rbm46-E14 cell colonies were much smaller than those formed by pPE-E14 cells (Fig 1C). Consistent with this observation, cell proliferation assays revealed a slower rate of proliferation in pPy-Rbm46-E14 cells (Fig 1B), suggesting Rbm46 has an inhibitory effect on ESC proliferation. The FACS results excluded the possibility that this effect is caused by apoptosis (Fig 1D).

**Fig 1:** Rbm46 inhibits mESC proliferation. (A) RT-PCR and Western Blot analysis of the pPy-Rbm46-E14 stable cell lines. (B) CCK-8 analysis of the proliferation rate of pPE-E14 cells and pPy-Rbm46 cells within 72 hours after seeding. Experiment was performed in triplicate. Error bars showed the standard deviation. (C) Statistics analysis of the average diameter of the colonies formed by pP-E14 cells and pPy-Rbm46 cells, respectively. Experiment was performed in triplicate. Error bars showed the standard deviation. ***, p<0.001; t-test. (D) Representative profiles of the pPE-E14 cells and pPy-Rbm46 cells by Annexin V/PI staining. (E) and (F) RT-PCR analysis of *Oct4* and *Rbm46* mRNA level at the indicated time points in E14 cells induced to undergo differentiation by removal of LIF. Experiments were performed in triplicate. Error bars showed the standard deviation.

We next evaluated expression levels of Rbm46 during mESC differentiation. mESCs were induced to differentiate by removal of LIF [14], and mRNA levels of *Oct4* and *Rbm46* were evaluated with qPCR. *Oct4* mRNA levels were significantly decreased (Fig 1E), while the *Rbm46* mRNA level showed a marked increase beginning on day 2 upon differentiation induction, and then decreased after day 6 (Fig 1F). The mRNA level of *Rbm46* was inversely correlated with that of Oct4, suggesting Rbm46 has a potential role in the regulation of mESC differentiation.

### Overexpression of Rbm46 results in differentiation of mESCs into trophectoderm

As we found endogenous Rbm46 was highly expressed during the process of mESC differentiation, we evaluated the influence of ectopic Rbm46 on mESC differentiation. We performed an alkaline phosphatase (AKP) staining analysis to detect the undifferentiated ESCs and found that pPE-E14 cells were almost 100% AKP positive (Fig 2B), and closely compacted (Fig 2A), a typical morphology of mESCs. In contrast, pPy-Rbm46-E14 cells were barely stained with AKP and grew in a loosely flat shape (Fig 2A). Moreover, immunostaining showed that the stem cell marker SSEA1 was strongly expressed in pPE-E14 cells, but not in pPRbm46-E14 cells (Fig 2A). FACS analysis showed that the percentage of SSEA1 positive pPE-E14 cells was higher than that of the SSEA1 positive pPy-Rbm46-E14 cells (79.07% vs 58.86%) (Fig 2B). These findings show Rbm46 promotes mESC differentiation. Teratocarcinoma formation is a tool for monitoring pluripotency in stem cell [21]. Subsequent experiment showed that teratocarcinoma formed by pPy-Rbm46-E14 cells was much smaller (by weight) than that formed by pPE-E14 cells (Fig 2C and 2D), suggesting Rbm46 compromised the ability of mESCs to form teratocarcinoma and possibly promoted differentiation.

**Fig 2:** Overexpression of Rbm46 results in differentiation of mESC into trophectoderm. (A) Left panel shows the morphology of the pPE-E14 cells and pPy-Rbm46 cells. Middle panel shows the AKP staining and immunostaining with SSEA-1 antibody of the pPE-E14 cells and pPy-Rbm46 cells. (B) FACs analysis of the SSEA-1 positive cells in pPE-E14 cells and pPy-Rbm46 cells. (C) and (D) Representative images and tumor weight analysis of the teratocarcinoma formed by pPE-E14 cells and pPRbm46 cells. (E) RT-PCR analysis of mRNA level of the marker from different layers in pPE-E14 cells and pPy-Rbm46 cells. The columns show the quantification of the indicated *gene* relative to *Gapdh*. The average value in the control group is normalized as 1. Experiment was performed in triplicate. Error bars showed the standard deviation. *, p<0.05; **, p<0.01, t-test. (F) RT-PCR analysis of the trophectoderm markers expressed in the teratocarcinoma formed by pPy-Rbm46 cells. The columns show the quantification of the indicated *gene* relative to *Gapdh*. The average value in the control group is normalized as 1. Experiment was performed in triplicate. Error bars showed the standard deviation. *, p<0.05, t-test.

We next asked what effect overexpression of Rbm46 would have on differentiation of mESCs. RT-PCR analysis showed that although there was no change in expression levels of markers for ectoderm (*Nestin*, *Glast*, *Notch*, *Neurogenin* and *Pax6*), mesoderm (*Brachyury*, *Bmp4*, *Nkx2*.*5*, *Myf5*, *MyoD*, *Adam19* and *Ephx2*) or endoderm (*Gata4*, *Gata6*, *Sox7*, *Sox17* and *Lama1*), overexpression of Rbm46 significantly elevated the mRNA level of the trophectoderm markers (*Cdx2*, *Eomes* and *Hand1*) (Fig 2E). RT-PCR analysis of the teratocarcinoma formed by pPy-Rbm46-E14 cell also showed an increase in the trophectoderm markers (*Cdx2* and *Eomes*) (Fig 2F). These results demonstrate that overexpression of Rbm46 promotes differentiation of mESCs into trophectoderm.

### *Rbm46* Knock-down promotes differentiation of mESCs into endoderm

We next investigated the influence of Rbm46 knock-down on mESC differentiation. We first established the *Rbm46* shRNA stable cell line that can effectively reduce the mRNA and protein level of Rbm46 (Fig 3A). Knock-down of Rbm46 promoted mESC differentiation, as suggested by the flat loosely shape morphology of the cells (Fig 3B). AKP staining and SSEA1 immuno-staining showed that mESCs silenced by Rbm46 is better differentiated, as defined by reduced level of SSEA1 and AKP staining signals (Fig 3B). In addition, FACS analysis showed that the percentage of SSEA1 positive cells was higher in the control group than in the *Rbm46* shRNA group (65.05% vs 49.82) (Fig 3C), and teratocarcinoma formed by *Rbm46*-silenced cells were much smaller in size and weight than those formed by the control cells (Fig 3D). These results indicated silencing of *Rbm46* compromises the ability of mESC to form teratocarcinoma and probably promotes mESC differentiation. Subsequent experiments also reflected the influence of deletion of *Rbm46 on* mESC differentiation. RT-PCR analysis showed that Rbm46 knock-down significantly increased the transcriptional level of endodermal markers (*Gata4*, *Gata6*, *Sox7*, *Sox17* and *Lama1*), while mRNA levels for markers of ectoderm (*Nestin*, *Glast*, *Notch*, *Neurogenin* and *Pax6*), mesoderm (*Brachyury*, *Bmp4*, *Nkx2*.*5*, *Myf5*, *MyoD*, *Adam19* and *Ephx2*) and trophectoderm (*Cdx2*, *Eomes* and *Hand1*) were unchanged (Fig 3E). RT-PCR analysis of the teratocarcinoma which resulted from *Rbm46*-silenced cells confirmed that *Rbm46* silencing significantly increased transcription of endodermal markers (*Gata6*, *Sox17* and *Lama1*) (Fig 3F). Our data indicate that silencing of Rbm46 promotes differentiation of mESCs into endoderm.

**Fig 3:** Downregulation of Rbm46 promotes differentiation of mESC into endoderm. (A) RT-PCR and Western Blot analysis of the *Rbm46* shRNA-E14 stable cell lines. (B) Left panel shows the morphology of the Non-silence cells and *Rbm46* shRNA cells. Middle panel shows the AKP staining and immunostaining with SSEA-1 antibody of Non-silence cells and *Rbm46* shRNA cells. (C) FACs analysis of the SSEA-1 positive cells in Non-silence cells and *Rbm46* shRNA cells. (D) and (E) Representative images and tumor weight analysis of the teratocarcinoma formed by Non-silence cells and *Rbm46* shRNA cells. (F) RT-PCR analysis of mRNA level of the marker from different layers in Non-silence cells and *Rbm46* shRNA cells. The columns show the quantification of the indicated *gene* relative to *Gapdh*. The average value in the Non-silence group is normalized as 1. Experiment was performed in triplicate. Error bars showed the standard deviation. *, p<0.05; **, p<0.01; ***, p<0.001; t-test. (G) RT-PCR analysis of the endoderm markers expressed in the teratocarcinoma formed by *Rbm46* shRNA cells. The columns show the quantification of the indicated *gene* relative to *Gapdh*. The average value in the Non-silence group is normalized as 1. Experiment was performed in triplicate. Error bars showed the standard deviation. *, p<0.05; ***, p<0.001; t-test.

### Rbm46 regulates mESC differentiation through down-regulation of *β-Catenin*

The Wnt- β-Catenin pathway is closely associated with maintenance of ESC pluripotency. Previous studies have shown that activation of the Wnt pathway stabilizes β-Catenin in the cytosol by releasing it from the destruction complex. Upon release, β-Catenin can translocate to the nucleus and activate the transcription of *Oct4* and *Rex1* [20, 22–24]. Among these factors, it is the level of OCT4 that determines whether ES cells differentiate into trophectoderm or endoderm [13, 25, 26]. In view of the fact that *Rbm46* RNA levels are inversely correlated with *Oct4* RNA levels during mESC differentiation, together with the fact that overexpression of Rbm46 or knock-down of *Rbm46* results in differentiation of mESCs into trophectoderm or endoderm respectively, we reasoned that Rbm46 may regulate mESC differentiation by acting on components of the Wnt pathway.

We first evaluated the influence of Rbm46 on the protein level of activated β-Catenin. Western blot showed that overexpression of Rbm46 significantly reduces both the protein and mRNA levels of total β-Catenin, activated β-Catenin, and Oct4 (Fig 4A and 4B), while knock-down of Rbm46 showed an inverse result (Fig 4C and 4D). However, Rbm46 had no influence on the protein level of GSK-3β (Fig 4A). GSK-3β is one of the critical components of the destruction complex for β-Catenin which can be inhibited by the Wnt signaling. Therefore, the influence of Rbm46 on β-Catenin does not rely on the GSK-3β activity. Lithium chloride (LiCl) has been shown to activate the Wnt/β-Catenin pathway [27]. Our results showed that LiCl not only elevated the protein level of active β-Catenin, but also rescued the reduced Oct4 caused by Rbm46 overexpression, suggesting that Oct4 is regulated by Rbm46 through downregulation of β-Catenin (Fig 4E). Further, while Rbm46 overexpression only caused mESC differentiation, as indicated by the loosely flat shape of the cells and the weak AKP staining, this effect was offset by treatment of LiCl to a large extent, indicating the influence of Rbm46 on mESC is associated with its regulation of β-Catenin (Fig 4F).

**Fig 4:** Rbm46 downregulates the mRNA level of *β-Catenin*. (A) pPE-E14 cells (Control) and pPy-Rbm46 cells were lysed and subjected to western blot with the indicated antibodies. (B) RT-PCR analysis of the indicated mRNA levels in pPE-E14 cells (Control) and pPy-Rbm46 cells. Experiment was performed in triplicate. Error bars showed the standard deviation. **, p<0.01; t-test. (C) Non-silence cells and *Rbm46* shRNA cells were lysed and subjected to western blot with the indicated antibodies. (D) RT-PCR analysis of the indicated mRNA levels in Non-silence cells and *Rbm46* shRNA cells. Experiment was performed in triplicate. Error bars showed the standard deviation. ***, p<0.001; t-test. (E) E14 cells were transfected with either empty vector or pPy-Rbm46 plasmid for 48 hours and treated with or without 10mM LiCl for 4 hours. The morphology and the AKP staining of the cell were viewed under microscope. (F) The cells treated as in (E) were lysed and subjected to western blot analysis with the indicated antibodies. (G) and (H) Luciferase reporter plasmid pGL3pro-3’UTR was transfected into Hela cells either with Rbm46 plasmid or Rbm46 plasmid plus *Rbm46* RNAi. Luciferase activities were measured after 48 h. The Luciferase activity was normalized to the control reporter (SV40 Poly A) activity. Experiments were performed in triplicate. Error bars showed the standard deviation. ***, p<0.001; t-test for (G) and one-way ANOVA with Tukey’s post hoc test for (H).

The RNA binding function of Rbm46 and its location in the cytoplasm (S2 Fig) indicates the possibility that Rbm46 may regulate β-Catenin by directly targeting its mRNA. As most cellular mRNAs are degraded primarily through the 3’ UTR polyA tail, we cloned the *β-Catenin* 3’ UTR polyA tail into the pGL3-promotor plasmid between the luciferase gene and SV40 polyA sequence (pGL3pro-3’UTR) (S3 Fig) and performed luciferase assays. Over-expression of Rbm46 reduced mRNA levels of *β-Catenin* 3’ UTR polyA in a dose-dependent manner by luciferase assay (Fig 4G), and this reduction was reversed by knockdown of Rbm46 (Fig 4H). These data suggested that Rbm46 targets the 3’ UTR of the *β-Catenin* mRNA.

### Rbm46 interacts with the P-bodies

To determine precisely how Rbm46 regulates β-Catenin, we overexpressed FLAG-Rbm46 in E14 and performed a FLAG IP. The immunoprecipitates were subjected to mass spectrum (MS) analysis. MS results showed that Rbm46 interacts with multiple proteins (Hnrnpu, Pabpc1, Igf2bp1, Ddx5, Hnrnpa1, Hnrnpa2b1, Sfrs1 and Rps19) which are critical effectors of post-transcriptional regulation (Fig 5A). In addition, *β-Catenin* mRNA could also be pulled down by Rbm46 (Fig 5B), suggesting *β-Catenin* mRNA directly interacts with the Rbm46 complex. Among the proteins pulled down by Rbm46, Pabpc1 (Poly A binding protein C1) which is a critical component of the P-bodies, is essential for mRNA degradation through the 3’ UTR polyA tail [28, 29]. We surmised Rbm46 interacts with Pabpc1 to degrade *β-Catenin* mRNA, and co-focal analysis showed that Rbm46 co-localizes with Pabpc1 in the cytoplasm (Fig 5C). Consistent with this finding, immunoprecipitation assay showed that ectopic Rbm46 interacted with endogenous Pabpc1 *in vivo* (S4 Fig). These data indicate that Rbm46 targets *β-Catenin* mRNA for degradation through interaction with the P-bodies.

**Fig 5:** Rbm46 interacts with the P-bodies. (A) pPy-Rbm26 cells which can stably express Flag-Rbm46 were lysed and subjected to FLAG immunoprecipitation, followed by MS analysis. (B) Flag-Rbm46 was transfected into E14 cells for 24 hours and were lysed and subjected to FLAG immunoprecipitation. Total RNA extracted from the eluate was subjected to RT-PCR with primers specific to *β-Catenin* and *Gapdh* (negative control). (C) Double immunofluorescence staining using antibodies against Rbm46 (red) and Pabpc1 (green) shows a clear co-localization in E14/T mESCs.

## Discussion

Our study reveals that Rbm46 is a critical regulator of ESC pluripotency based on changes observed in mESC differentiation under the influence of alterations in Rbm46. We first observed mRNA levels of *Rbm46* are markedly elevated during mESC differentiation. Subsequent experimental results showed that over-expression of Rbm46 leads to mESC differentiation into trophectoderm, while knock-down of Rbm46 promotes mESC endodermal differentiation. In addition, we found the mechanism by which Rbm46 regulate differentiation involves targeting of *β-Catenin* mRNA for degradation, which leads to decreased transcription of *Oct4*.

Stem cell pluripotency is regulated by a variety of transcription factors and multiple signaling pathways. Among these transcription factors, Oct4, Sox2 and Nanog have been identified as the most essential regulators of stem cell pluripotency [30]. These factors, together with signaling pathways such as the LIF/STAT3 and Wnt pathways form a complex network for regulation of stem cell pluripotency [3, 25, 31, 32]. The LIF/STAT3 was the first pathway identified as having the potential to maintain the pluripotency of mESC. Later, the Wnt pathway was found to have similar functions [15]. Both pathways regulate the transcription of *Oct4* [33, 34]. The transcriptional regulation of *Oct4* by these two pathways has been very extensively studied. However, little is known about the post-transcriptional regulation of *Oct4*.

In this study, we report a novel RNA binding protein RBM46 which is highly expressed in ESCs. A previous report showed that multiple RNA binding proteins (RBPs) are highly expressed in ESCs as compared with differentiated cells [8]. Some RBPs have been shown to regulate the pluripotency of stem cells [35]. These studies argue RBPs play a significant role in stem cell regulation. We show that overexpression of Rbm46 significantly inhibits mESC proliferation, and promotes mESC differentiation into trophectoderm. Silencing of *Rbm46* does not inhibit mESC differentiation, but enhances mESC differentiation into endoderm, suggesting Rbm46 regulates the machinery which is essential for ESC pluripotency. RBPs are proteins responsible for the control of RNA stability, processing, and translation [24], and we identified the target mRNA of Rbm46. Oct4 is transcriptionally activated by β-Catenin, and has been shown to determine the direction of ESC differentiation, and this molecule was downregulated by Rbm46 in our study. Overexpression of Rbm46 reduced the protein and mRNA levels of β-Catenin without affecting the GSK-3β level, suggesting regulation of β-Catenin by Rbm46 is Wnt independent. We demonstrated Rbm46 interacts with the P-bodies and directly targets *β-Catenin* mRNA for degradation through its 3’ UTR polyA tail.

The study reveals novel functions of Rbm46 and demonstrates the mechanism through which Rbm46 regulates *β-Catenin* mRNA stability and stem cell pluripotency. Our results reveal that Rbm46 is one of the important regulators of ESC pluripotency.

## Supporting information

S1 Fig Bioinformatics of *Rbm46*. (A) The sequence of *Rbm46* is highly conserved among different species. (B)Schematic figure of the RRM domains of *Rbm46*.
(TIF)

S2 Fig Localization of Rbm46. Immunofluorescence staining shows the localization of endogenous Rbm46 and ectopic Rbm46 (Flag-Rbm46) using antibodies against Rbm46 and Flag, respectively.
(TIF)

S3 Fig pGL3pro-3’UTR reporter plasmid information. Schematic illustration of the construction of pGL3pro-3’UTR reporter plasmid.
(TIF)

S4 Fig Rbm46 interacts with Pabpc1. pPE-E14 cells (Mock cells) and pPy-Rbm26 cells were lysed and subjected to Flag immunoprecipitation, followed by western blot with the indicated antibodies.
(TIF)

S1 Table Primers for RT-PCR. S1 Table shows the detailed sequence of the primers for RT-PCR.
(PDF)
